# Inflammatory cytokine‐mediated induction of serine racemase in atopic dermatitis

**DOI:** 10.1111/jcmm.13592

**Published:** 2018-03-22

**Authors:** Yoko Yoshihisa, Mati Ur Rehman, Maho Nakagawa, Shoko Matsukuma, Teruhiko Makino, Hisashi Mori, Tadamichi Shimizu

**Affiliations:** ^1^ Department of Dermatology Graduate School of Medicine and Pharmaceutical Sciences University of Toyama Toyama Japan; ^2^ Department of Radiology Graduate School of Medicine and Pharmaceutical Sciences University of Toyama Toyama Japan; ^3^ Advanced Technology Research Center FANCL Research Institute Yokohama Japan; ^4^ Department of Molecular Neuroscience Graduate School of Medicine and Pharmaceutical Sciences University of Toyama Toyama Japan

**Keywords:** atopic dermatitis, keratinization, serine racemase

## Abstract

Serine racemase (SR) is an enzyme that catalyses the synthesis of d‐serine, an endogenous coagonist for *N*‐methyl‐D‐aspartate (NMDA)‐type glutamate receptor in the central nervous system. Our previous study demonstrated that SR was expressed in the epidermis of wild‐type (WT) mice but not in SR knockout (KO) mice. In addition, SR immune‐reactivity was only found in the granular and cornified layers of the epidermis in WT mice. These findings suggested that SR is involved in the differentiation of epidermal keratinocytes and the formation of the skin barrier. However, its role in skin barrier dysfunction such as atopic dermatitis (AD) remains elusive. AD is a chronic inflammatory disease of skin, and the clinical presentation of AD has been reported to be occasionally associated with psychological factors. Therefore, this study examined the content of d‐serine in stratum corneum in AD patients and healthy controls using a tape‐stripping method. Skin samples were collected from the cheek and upper arm skin of AD patient's lesion and healthy individuals. The d‐serine content was significantly increased in the involved skin of AD in comparison with healthy individuals. An immunohistochemical analysis also revealed an increased SR expression in the epidermis of AD patients. Furthermore, the SR expression in cultured human keratinocytes was significantly increased by the stimulation with tumour necrosis factor ‐α or macrophage migration inhibitory factor. Taken together, these findings suggest that d‐serine expressed particularly strongly in AD lesional skin and that the SR expression in the keratinocytes is linked to inflammatory cytokines.

## 1 INTRODUCTION

In the central nervous system (CNS), d‐serine, an endogenous coagonist for *N*‐methyl‐D‐aspartate (NMDA)‐type glutamate receptor, is catalysed by the biosynthetic enzyme serine racemase (SR), which is involved in the conversion of l‐serine into d‐serine.^1^ NMDA receptor is an ionotropic glutamate receptor, which plays a major role in the CNS. Its activation is regulated by excitatory neurotransmitter, glutamate, to perform essential functions responsible in controlling synaptic plasticity in the course of learning and memory formation.^2^, ^3^ d‐Serine, an endogenous NMDA receptor coagonist, is widely distributed in the CNS and thought to potentiate the activity of NMDA receptor. Indeed, its depletion can inhibit NMDA receptor‐mediated neurotransmission.^4^, ^5^, ^6^ The immune cells and keratinocytes are reported to be directly affected by psychological factor‐induced biochemical changes in the brain and peripheral nervous system.^7^ Recent studies have shown that the NMDA receptor is expressed in the human epidermis in addition to the CNS, and the activation of the NMDA receptor was found to inhibit the process of re‐epithelization.^8^, ^9^

It has been shown that amyloid β peptide (Aβ) and lipopolysaccharide stimulation can induce the expression of SR from microglia. It was noted that the elevation of SR is linked to the increases in the steady‐state level of SR mRNA.^10^, ^11^ In addition, SR expression was also reported in peripheral nerve‐derived Schwann cells and fibroblasts.^12^ These findings suggest that the induction of SR expression following pro‐inflammatory stimulation highlights the important connection between neuro‐inflammation and excitotoxicity.^10^, ^11^ Atopic dermatitis (AD) is a chronic inflammatory disease of skin, characterized by infiltration of inflammatory cells, itching, and a clinical course representative of symptomatic flares and remissions. While the exact underlying mechanism in AD pathogenesis remains elusive, the clinical presentation of AD has occasionally been linked to psychological factors. Our previous study postulated SR protein localization in the granular and cornified epidermal layer of mice and its presence in keratinocytes.^13^ However, the role of the SR in the inflammatory phase in AD remains elusive. Therefore, we examined the expression of SR in AD patients’ skin and its association with inflammatory cytokines.

## 2 MATERIALS AND METHODS

### 2.1 Reagents

A keratinocyte growth medium (KGM) was purchased from Kurabo Industries, Ltd. (Osaka, Japan). The nylon membranes were obtained from Millipore (Bedford, MA, USA). Recombinant human interleukin (IL)‐4, IL‐5, tumour necrosis factor (TNF)‐α, macrophage migration inhibitory factor (MIF), and IL‐1β were ordered from R&D Systems (Minneapolis, MN, USA). The antiserine racemase (ab123894) monoclonal antibody was from Abcam (Cambridge, MA, USA), and anti‐β‐actin antibody was from Sigma‐Aldrich Co (St. Louis, MO, USA). The detection system for Western blot was purchased from Cell Signaling Technology (Beverly, MA, USA). The other reagents used in the study were of analytical grade.

### 2.2 Patients and the evaluation of clinical features

Twenty AD patients (13 males and 7 females; mean age, 31.1 years [range, 20‐44 years]) were included in this study. The patients were diagnosed with AD according to the criteria of Hanifin and Rajka. No other associated disease was present in patients. In addition, nineteen healthy control individuals (11 males and 8 females; mean age, 37.2 years [range, 29‐55 years]) without any prior history of atopic disease were also enrolled. The study was approved by the Ethics Committee of the University of Toyama.

### 2.3 Tape‐stripping of the stratum corneum

Tape‐stripping method was employed to obtain samples from stratum corneum (SC) using skin tape (Harney Layer Checker; Asahi Biomed, Tokyo, Japan). The tape was placed over a skin lesion on AD patients’ cheeks as ultraviolet (UV) exposed area or upper arms as UV un‐exposed area and carefully pressed with a finger before being pulled away. Similarly, control SC samples were taken from a nearby area of uninvolved skin in AD patients as well as from healthy individuals. The SC samples were extracted from the tape strips by ultrasonication with 500 μL of PBS (phosphate‐buffered saline) containing 0.05% Tween 20. After mixing in a vortex mixer, the extract aliquots were placed into vials and stored at −80°C.

### 2.4 Measurement of d‐serine and l‐serine

Reverse‐phase high‐performance liquid chromatography (HPLC) was used to separate and detect d‐serine and l‐serine in samples.^14^ Samples were extracted using an 85:15 mixture of perchloric acid aqueous solution (pH 1.5):acetonitrile. The extraction liquid was analysed for d‐serine and l‐serine concentrations by HPLC (Shimadzu HPLC Amino Acid Analysis System, Shimadzu Corporation, Kyoto, Japan) using a post‐column derivatization method. The CROWNPAK CR‐I (+) column (3 mm id × 150 mm; Daicel Corporation, Tokyo, Japan) was used as the HPLC column in a container cooled below 0°C during the analysis. Fluorescence was monitored with 344 nm excitation and 443 nm emission. The contents of l‐ and d‐serine were expressed as ng/μg protein.

### 2.5 Cell culture and treatments

Normal human epidermal keratinocytes (NHKs; Kurabo Industries Ltd.) were cultured in KGM containing epidermal growth factor (0.1 ng/mL), insulin (5 and 10 μg/mL), hydrocortisone (0.5 μg/mL), bovine pituitary extract (0.4%), gentamicin (50 μg/mL), and amphotericin B (50 ng/mL) at 37°C in 5% CO_2_ in air. All experiments were carried out on cells at the third or fourth passages, when cells reached to 90% confluency, they were subjected to analysis. The concentration of cytokines in keratinocytes stimulation experiments was decided based on their basal circulating level according to our previous study. MIF basal circulating levels are 1000‐fold higher than other cytokines. In the relevant experiments, IL‐4 (0‐1000 pg/mL), IL‐5 (0‐1000 pg/mL), TNF‐α (0‐1000 pg/mL), IL‐1β (0‐1000 pg/mL), or MIF (0‐100 ng/mL) was added. Our preliminary experiments showed no toxicity for keratinocytes at each concentration of cytokines. Samples were obtained 48 hours after an addition of cytokines.

### 2.6 Western blot analyses

The human skin specimens were homogenized using a Polytron homogenizer (Kinematica, Lausanne, Switzerland). After homogenization, skin or cells were collected and rinsed in cold PBS, and then lyses were performed in RIPA buffer for 10 minutes. Following brief sonication, the cell lysates were centrifuged at a speed of 13 200 g for 10 minutes at 4°C. Then the measurement of protein content in supernatants was performed with a Bio‐Rad Protein Assay kit (Bio‐Rad, Hercules, CA, USA). After mixing with SDS‐loading buffer, denaturation of protein lysates was done by heating at 96°C for 5 minutes. Finally, the protein lysates were loaded for electrophoresis to an SDS polyacrylamide gel and transferred to nylon membranes. A Western blot analysis was carried out to detect the expression of serine racemase using an antibody. Band signals were visualized using ECL Plus detection reagent (GE Healthcare, Waukesha, WI, USA), and then the luminescent signals were evaluated using LAS‐4000 (Fujifilm, Tokyo, Japan). β‐actin was used as an internal control to normalize the relative amounts of SR.

### 2.7 Immunohistochemistry of skin

Human skin tissue samples were immersed into OCT Compound (Ted Pella, Redding, CA, USA) and then frozen using liquid nitrogen. Sections measuring 5 μm in thickness were blocked with Protein Block Serum‐Free (DAKO, Carpentaria, CA, USA) for 30 minutes and then incubated with the primary antibodies. Sections were then rinsed with PBS and immunoreacted with biotinylated goat antimouse IgG (Bector) for 30 minutes. The signals were detected with Envision+ (DAKO), followed by staining using the Liquid DAB+ Substrate Chromogen System (DAKO). The nuclei were counterstained with haematoxylin. The tissue sections were observed using a microscope (Nikon, Tokyo, Japan).

### 2.8 Immunocytochemistry of cultured cells

Cultured cells were washed with PBS and then fixed using 4% paraformaldehyde in PBS for 1 hour at room temperature. Following fixation, cells were again rinsed in PBS and blocked with Protein Block Serum‐Free for 30 minutes. After blocking, cells were exposed to primary anti‐SR antibody for 1 hour at 4°C, and then treated with FITC‐conjugated antimouse IgG (MBL) for 1 hour at room temperature. Finally, the samples were analysed under a fluorescence microscope (Olympus, Tokyo, Japan).

### 2.9 Statistical analysis

The statistical differences between the test and control groups were analysed using either Student's *t* test or one‐way analysis of variance. Data are shown as the means ± standard deviation (SD).

## 3 RESULTS

### 3.1 Measurement of l‐serine and d‐serine contents in the SC of AD patients and healthy controls

To confirm the presence of l‐ and d‐serine in the SC of AD patients and healthy controls, reverse‐phase HPLC was performed. Symptoms of AD are occasionally aggravated by exposure to environmental hazards or UV exposure. To exclude an effect of environmental hazards or UV exposure in a production of l‐serine or d‐serine, the stratum corneum samples were obtained both from AD patient's cheek as UV exposed area and from upper arm as UV un‐exposed area. The results showed that the l‐serine content in AD‐involved and uninvolved skin samples was significantly lower than that in healthy control samples (*P* < .005 vs *P* < .001 for cheek samples and *P* < .001 for upper arm samples), while the d‐serine content was significantly higher than that in healthy control samples (*P* < .05 vs *P* < .01 for both the cheek and the upper arm). In addition, cheek and upper arm samples from AD skin also showed significantly higher d‐form ratios than did healthy control (*P* < .005, *P* < .001, and *P* < .05, respectively) (Figure 1).

**Figure 1:** The stratum corneum d‐serine, l‐serine, and d‐form levels in AD patients and healthy controls. The d‐serine and l‐serine contents (ng/μg protein) were measured in the stratum corneum samples obtained from the involved and uninvolved areas in AD patients (n = 20) and normal healthy controls (n = 19). A, Cheek, B, Upper arm. The Steel‐Dwass test was used to compare the d‐serine and l‐serine levels between the AD patients and healthy control individuals. The data are expressed as the mean ± standard deviation of the mean

### 3.2 SR expression in the epidermis of AD and healthy controls

d‐Serine is mainly produced by conversion from l‐serine via the action of SR. We next examined the SR expression in AD‐involved skin to determine the correlation of SR with d‐serine in the SC. An immunohistochemical analysis was done using skin samples from healthy control and AD involved with high d‐serine content. The expression of SR was markedly observed in the upper spinous, granular, and horny layers of the AD‐involved skin samples in comparison with those in healthy controls (Figure 2A). We also examined the SR protein expression in the epidermis of AD‐involved skin samples and healthy controls by a Western blot analysis. The signal of SR protein was substantially higher in the epidermis of AD‐involved skin samples than in healthy controls (Figure 2B).

**Figure 2:** Expression of SR in AD patients’ involved skin and healthy controls. A, Immunohistochemical staining of AD patients’ involved skin and healthy control skin with anti‐SR antibody. SR immune‐reactivity was observed in the epidermis of AD patients but not in the healthy controls. Scale bar = 100 μm. (a)‐(c) upper panel AD patients, lower panel on higher magnification; (d) upper panel healthy controls, lower panel on higher magnification. B, A Western blot analysis of SR protein in AD patients’ involved skin and healthy controls using anti‐SR and anti‐actin antibodies

### 3.3 Effects of inflammatory cytokines on the SR protein expression in cultured keratinocytes

Inflammatory cytokines are known to play a crucial role in the pathogenesis of AD. There is growing evidence to suggest that Th2 cytokines adversely affect the skin barrier function. Therefore, the relationship between Th2 cytokines, including IL‐4, IL‐5, and pro‐inflammatory cytokines (TNF‐α, MIF, and IL‐1β), and SR protein was examined in cultured keratinocytes at 90% confluency by a Western blot analysis. Upon stimulation with IL‐4, IL‐5, and IL‐1β, the SR expression was not increased even at higher concentration. However, the SR expression was significantly and dose‐dependently increased on stimulation with TNF‐α or MIF (Figure 3A). Especially, stimulation with MIF abundantly induced SR. For further confirmation, TNF‐α and MIF were chosen for immunofluorescence staining of SR in cultured confluent keratinocytes. Consistent with the findings of Western blot analysis, immunofluorescence staining also showed increased SR expression with TNF‐α and MIF, with the SR expression markedly increased on MIF treatment (Figure 3B).

**Figure 3:** Correlation of SR with inflammatory cytokines in cultured 90% confluency keratinocytes. A, A Western blot analysis of SR protein in the presence of Th‐2 cytokines ((a) IL‐4 (0‐1000 pg/mL), (b) IL‐5 (0‐1000 pg/mL)) and pro‐inflammatory cytokines ((c) TNF‐α (0‐1000 pg/mL), (d) IL‐1β (0‐1000 pg/mL) and (e) MIF (0‐100 ng/mL)) using anti‐SR and anti‐actin antibodies. β‐Actin was used to normalize the expression level. Band densities were measured using ImageJ software to evaluate the intensity of bands. Quantitative data obtained from 3 independent experiments are presented. B, Immunofluorescence staining of SR (green) in the presence of TNF‐α (1000 pg/mL) and MIF (100 ng/mL). Nuclei were counterstained with 4′,6‐diamidino‐2‐phenylindole (DAPI, blue). Scale bar = 100 μm

## 4 DISCUSSION

Skin, the outermost layer of the body, is continuously exposed to environmental stresses. Skin is also supplied by a cutaneous network of sensory fibres, and similar neurotransmitters and neuropeptide receptors to those found in the CNS are expressed in the skin.^7^, ^15^ Furthermore, skin plays a crucial role in bidirectional crosstalk between the immune, nervous, and endocrine systems by regulating several biochemical mediators. Aberrant regulation of such biochemical mediators in the CNS and skin has been linked to the AD pathophysiology.^16^, ^17^

In this study, we examined for the first time the content of l‐serine and d‐serine in the SC of the skin of AD patients. The content of d‐serine was markedly higher in the involved skin lesions than in the uninvolved skin lesion and in SC samples of healthy individuals. Furthermore, increased expression of SR was detected in the epidermis of AD‐involved skin samples in comparison with those in healthy individuals. d‐Serine is known to act as an endogenous NMDA receptor coagonist in the CNS.^4^, ^5^, ^6^ Recent study has shown that the NMDA receptor is expressed in the epidermis of human skin, and the activation of the NMDA receptor was found to influence the keratinocyte proliferation, differentiation, and migration during epithelization.^9^ The exact function of d‐serine in keratinocytes remains elusive; however, we suggest that d‐serine might act as a coagonist of the NMDA receptor in human keratinocytes.

We next examined the relationship between inflammatory cytokines and the SR expression using cultured keratinocytes. The SR expression was found to be increased following stimulation with MIF and TNF‐α, with the increase observed after MIF treatment being more profound. In AD skin lesions, inflammatory cytokines and growth factors, like IL‐4, IL‐5, IL‐6, TNF‐α, and granulocyte macrophage colony‐stimulating factor, have been reported to be produced and associated with the pathogenesis of AD.^18^ In addition, our previous studies found that the expression of MIF was increased in AD patients’ skin keratinocytes^19^ and peripheral blood mononuclear cells.^20^ Furthermore, we previously demonstrated that the MIF level in the SC samples obtained from the cheek, neck, and upper arm areas of the involved skin of AD patients was closely associated with the lesion severity.^21^ Therefore, the findings of the present study suggest a positive correlation between the MIF and SR expression. Given these findings, we suggested that inflammatory cytokines, specifically MIF, might induce SR expression in the involved skin of AD patients.

We recently showed that SR protein is present in the epidermis of WT mice but not in the SR knockout (KO) mice and described a mechanism for l‐serine to d‐serine conversion in epidermal keratinocytes, suggesting the role of SR in epidermal keratinocytes differentiation and skin barrier formation.^13^ Considering the findings of our previous study, we expected that the d‐serine content would be decreased because of AD‐induced skin barrier disruption. However, in contrast, this study showed increased d‐serine content in AD patients’ involved skin samples. The reason for this is that in our previous study, the experiments were performed using SR KO mice; therefore, a similar role of SR in human skin cannot be expected because of species differences between humans and mice, which will need to be evaluated in future studies.

In conclusion, the result presented in this study showed that d‐serine levels in SC in the cheek and upper arm skin were positively related to the local skin lesion. In addition, SR expression in AD‐involved skin is associated with inflammatory cytokines especially MIF. Therefore, it can be speculated that detection of d‐serine in combination with MIF in SC would become an effective strategy to assess the local skin lesion in AD patients. Although SR and d‐serine exact function in human skin still awaits further investigation, however, their roles in skin inflammation are not negligible. In future, development of agents blocking d‐serine production might be beneficial to control inflammation in AD patients.
